# Tetra-μ-2,5-difluoro­benzoato-bis­[(2,2′-bipyridine)(2,5-difluoro­benzoato)gadolinium(III)]

This article has been retracted.

**DOI:** 10.1107/S1600536808023507

**Published:** 2008-08-09

**Authors:** Sheng Li, Fu-Li Zhang, Kun Tang, Yuan-Fang Ma

**Affiliations:** a The Institute of Immunology, Key Laboratory of Natural Drugs and Immunological Engineering of Henan Province, College of Medicine, Henan University, Kaifeng 475003, People’s Republic of China; b College of Medicine, Henan University, Kaifeng 475003, People’s Republic of China

## Abstract

In the centrosymmetric title compound, [Gd_2_(C_7_H_3_F_2_O_2_)_6_(C_10_H_8_N_2_)_2_], the asymmetric unit comprises one cation chelated by two 2,5-difluoro­benzoate and one 2,2′-bipyridine. Two cations are linked into dimers *via* three bridging carboxyl­ate groups from three 2,5-difluoro­benzoic acid units. The Gd^III^ ion is nine-coord­inated by seven O atoms and two N atoms.

## Related literature

For related literature, see: Church & Halvorson (1959 ▶); Chung *et al.* (1971 ▶); Okabe & Oya (2000 ▶); Okabe *et al.* (2002 ▶); Serre *et al.* (2005 ▶); Pocker & Fong (1980 ▶); Scapin *et al.* (1997 ▶).

## Experimental

### 

#### Crystal data

[Gd_2_(C_7_H_3_F_2_O_2_)_6_(C_10_H_8_N_2_)_2_]
*M* *_r_* = 1569.43
Triclinic,
*a* = 11.4012 (10) Å
*b* = 12.1890 (10) Å
*c* = 12.588 (2) Å
α = 103.99 (2)°
β = 102.90 (2)°
γ = 113.58 (2)°
*V* = 1451.6 (3) Å^3^
*Z* = 1
Mo *K*α radiation
μ = 2.37 mm^−1^
*T* = 293 (2) K
0.44 × 0.26 × 0.20 mm

#### Data collection

Bruker APEXII CCD area-detector diffractometer
Absorption correction: multi-scan (*SADABS*; Bruker, 2001 ▶) *T*_min_ = 0.422, *T*_max_ = 0.648
8233 measured reflections
5557 independent reflections
4813 reflections with *I* > 2σ(*I*)
*R*_int_ = 0.021

#### Refinement

*R*[*F* ^2^ > 2σ(*F* ^2^)] = 0.041
*wR*(*F* ^2^) = 0.110
*S* = 1.00
5557 reflections
416 parameters
H-atom parameters constrained
Δρ_max_ = 2.22 e Å^−3^
Δρ_min_ = −0.62 e Å^−3^

### 

Data collection: *APEX2* (Bruker, 2004 ▶); cell refinement: *SAINT-Plus* (Bruker, 2001 ▶); data reduction: *SAINT-Plus*; program(s) used to solve structure: *SHELXS97* (Sheldrick, 2008 ▶); program(s) used to refine structure: *SHELXL97* (Sheldrick, 2008 ▶); molecular graphics: *SHELXTL* (Sheldrick, 2008 ▶); software used to prepare material for publication: *SHELXTL*.

## Supplementary Material

Crystal structure: contains datablocks I, global. DOI: 10.1107/S1600536808023507/er2055sup1.cif

Structure factors: contains datablocks I. DOI: 10.1107/S1600536808023507/er2055Isup2.hkl

Additional supplementary materials:  crystallographic information; 3D view; checkCIF report

## supplementary crystallographic information

### Comment

In recent years, carboxylic acids have been widely used as polydentate ligands, which can coordinate to transition or rare earth ions yielding complexes with interesting properties that are useful in materials science (Church & Halvorson, 1959; Chung *et al.*, 1971) and in biological systems (Okabe & Oya, 2000; Serre *et al.*, 2005; Pocker & Fong, 1980; Scapin *et al.*, 1997). Herein, we report the synthesis and X-ray crystal structure analysis of the title compound, hexa(2,5-difluorobenzoato) bis(2,2'-bipyridine) bisgadolinium(III).

The molecular structure of the title compound is shown in Fig.1, Gd^III^ is chelated by two 2,5-difluorobenzoate and one 2,2'-bipyridine. Two cations are linked into a dimer *via* bridging carboxylate groups from four 2,5-difluorobenzoate ions. The Gd^III^ ion is nine-coordinated with seven O atoms and two N atoms. The Gd—N and Gd—O bond lengths are in the range of 2.567 (4)–2.585 (5) Å and 2.364 (4)–2.495 (4) Å, respectively.

### Experimental

A mixture of gadolinium chloride (0.5 mmol), 2,5-difluorobenzoic acid (1 mmol), Sodium hydroxide(1 mmol), 2,2'-bipyridine(0.5 mmol), H_2_O (8 ml) and Ethanol (8 ml) in a 25 ml Teflon-lined stainless steel autoclave was kept at 433 K for three days. Colorless crystals were obtained after cooling to room temperature.

### Refinement

All H atoms on C atoms were generated geometrically and refined as riding atoms with C—H= 0.93Å and *U*_iso_(H)= 1.2 times *U*_eq_(C).

### Crystal data

**Table:**

[Gd_2_(C_7_H_3_F_2_O_2_)_6_(C_10_H_8_N_2_)_2_]	*Z* = 1
*M**_r_* = 1569.43	*F*_000_ = 766
Triclinic, *P*1	*D*_x_ = 1.795 Mg m^−^^3^
Hall symbol: -P 1	Mo *K*α radiation λ = 0.71073 Å
*a* = 11.4012 (10) Å	Cell parameters from 5557 reflections
*b* = 12.1890 (10) Å	θ = 1.8–26.0º
*c* = 12.588 (2) Å	µ = 2.37 mm^−^^1^
α = 103.99 (2)º	*T* = 293 (2) K
β = 102.90 (2)º	Block, colorless
γ = 113.58 (2)º	0.44 × 0.26 × 0.20 mm
*V* = 1451.6 (3) Å^3^	

### Data collection

**Table:**

Bruker APEXII CCD area-detector diffractometer	5557 independent reflections
Radiation source: fine-focus sealed tube	4813 reflections with *I* > 2σ(*I*)
Monochromator: graphite	*R*_int_ = 0.021
*T* = 293(2) K	θ_max_ = 26.0º
φ and ω scans	θ_min_ = 1.8º
Absorption correction: multi-scan(SADABS; Bruker, 2001)	*h* = −10→14
*T*_min_ = 0.422, *T*_max_ = 0.649	*k* = −15→12
8233 measured reflections	*l* = −15→14

### Refinement

**Table:**

Refinement on *F*^2^	Secondary atom site location: difference Fourier map
Least-squares matrix: full	Hydrogen site location: inferred from neighbouring sites
*R*[*F*^2^ > 2σ(*F*^2^)] = 0.041	H-atom parameters constrained
*wR*(*F*^2^) = 0.110	*w* = 1/[σ^2^(*F*_o_^2^) + (0.071*P*)^2^ + 0.5036*P*] where *P* = (*F*_o_^2^ + 2*F*_c_^2^)/3
*S* = 1.00	(Δ/σ)_max_ = 0.030
5557 reflections	Δρ_max_ = 2.22 e Å^−^^3^
416 parameters	Δρ_min_ = −0.62 e Å^−^^3^
Primary atom site location: structure-invariant direct methods	Extinction correction: none

### Special details

**Table:**

Geometry. All e.s.d.'s (except the e.s.d. in the dihedral angle between two l.s. planes) are estimated using the full covariance matrix. The cell e.s.d.'s are taken into account individually in the estimation of e.s.d.'s in distances, angles and torsion angles; correlations between e.s.d.'s in cell parameters are only used when they are defined by crystal symmetry. An approximate (isotropic) treatment of cell e.s.d.'s is used for estimating e.s.d.'s involving l.s. planes.
Refinement. Refinement of *F*^2^ against ALL reflections. The weighted *R*-factor *wR* and goodness of fit *S* are based on *F*^2^, conventional *R*-factors *R* are based on *F*, with *F* set to zero for negative *F*^2^. The threshold expression of *F*^2^ > σ(*F*^2^) is used only for calculating *R*-factors(gt) *etc*. and is not relevant to the choice of reflections for refinement. *R*-factors based on *F*^2^ are statistically about twice as large as those based on *F*, and *R*- factors based on ALL data will be even larger.

### Fractional atomic coordinates and isotropic or equivalent isotropic displacement parameters (Å^2^)

**Table:**

	*x*	*y*	*z*	*U*_iso_*/*U*_eq_	
Gd1	0.39616 (2)	0.80450 (2)	0.43978 (2)	0.03327 (12)	
C1	0.5204 (7)	0.6201 (6)	0.2986 (6)	0.0566 (16)	
H1	0.5606	0.6949	0.2835	0.068*	
C2	0.5504 (8)	0.5214 (7)	0.2568 (7)	0.071 (2)	
H2	0.6112	0.5310	0.2168	0.086*	
C3	0.4902 (9)	0.4138 (7)	0.2755 (7)	0.074 (2)	
H3	0.5067	0.3456	0.2468	0.089*	
C4	0.4041 (8)	0.4025 (6)	0.3367 (6)	0.067 (2)	
H4	0.3630	0.3274	0.3511	0.080*	
C5	0.3784 (6)	0.5033 (5)	0.3773 (5)	0.0470 (15)	
C6	0.6740 (5)	0.9487 (5)	0.6191 (5)	0.0369 (11)	
C7	0.8263 (6)	1.0068 (5)	0.6801 (5)	0.0424 (13)	
C8	0.9145 (7)	1.0683 (6)	0.6300 (7)	0.0626 (18)	
H8	0.8813	1.0778	0.5601	0.075*	
C9	1.0543 (8)	1.1162 (7)	0.6852 (9)	0.079 (2)	
C10	1.1059 (8)	1.1078 (8)	0.7849 (9)	0.088 (3)	
H10	1.2004	1.1430	0.8197	0.105*	
C11	1.0194 (8)	1.0459 (9)	0.8400 (8)	0.084 (3)	
H11	1.0547	1.0395	0.9110	0.100*	
C12	0.8802 (6)	0.9953 (7)	0.7841 (6)	0.0538 (15)	
C13	0.1577 (6)	0.6867 (5)	0.2396 (5)	0.0403 (12)	
C14	0.0390 (6)	0.6516 (5)	0.1350 (5)	0.0457 (13)	
C15	−0.0965 (7)	0.5954 (7)	0.1250 (6)	0.0602 (17)	
C16	−0.2024 (7)	0.5661 (9)	0.0290 (7)	0.079 (2)	
H16	−0.2919	0.5269	0.0273	0.094*	
C17	−0.1783 (8)	0.5937 (8)	−0.0639 (7)	0.077 (2)	
H17	−0.2498	0.5751	−0.1299	0.092*	
C18	−0.0444 (9)	0.6503 (8)	−0.0579 (6)	0.074 (2)	
C19	0.0612 (7)	0.6787 (6)	0.0364 (6)	0.0595 (17)	
H19	0.1501	0.7167	0.0365	0.071*	
C20	0.6082 (5)	0.9901 (5)	0.3314 (5)	0.0379 (11)	
C21	0.6108 (6)	0.9679 (5)	0.2087 (5)	0.0440 (13)	
C22	0.7087 (7)	1.0531 (6)	0.1808 (6)	0.0552 (16)	
C23	0.7022 (9)	1.0268 (7)	0.0655 (7)	0.068 (2)	
H23	0.7709	1.0843	0.0480	0.082*	
C24	0.5951 (9)	0.9165 (8)	−0.0237 (7)	0.0695 (19)	
H24	0.5889	0.9002	−0.1014	0.083*	
C25	0.5001 (8)	0.8335 (7)	0.0047 (6)	0.0660 (18)	
C26	0.5039 (6)	0.8539 (6)	0.1199 (6)	0.0528 (15)	
H26	0.4374	0.7935	0.1369	0.063*	
C27	0.2142 (7)	0.6084 (7)	0.5643 (7)	0.0621 (18)	
H27	0.2169	0.6855	0.6019	0.075*	
C28	0.1338 (8)	0.5019 (8)	0.5805 (8)	0.078 (2)	
H28	0.0841	0.5069	0.6292	0.094*	
C29	0.1264 (9)	0.3904 (8)	0.5264 (9)	0.091 (3)	
H29	0.0694	0.3160	0.5350	0.109*	
C30	0.2040 (9)	0.3852 (7)	0.4569 (8)	0.084 (3)	
H30	0.2005	0.3077	0.4192	0.101*	
C31	0.2871 (6)	0.4973 (5)	0.4440 (5)	0.0527 (16)	
F1	0.8152 (5)	1.1601 (4)	0.2644 (4)	0.0831 (13)	
F2	0.3947 (6)	0.7242 (5)	−0.0810 (4)	0.1036 (18)	
F3	0.7955 (5)	0.9343 (6)	0.8322 (4)	0.0982 (17)	
F4	1.1395 (6)	1.1740 (7)	0.6349 (8)	0.139 (3)	
F5	−0.1314 (7)	0.5674 (10)	0.2087 (7)	0.179 (4)	
F6	−0.0098 (10)	0.6785 (11)	−0.1474 (8)	0.217 (5)	
N1	0.2898 (5)	0.6091 (4)	0.4975 (5)	0.0485 (12)	
N2	0.4380 (5)	0.6129 (4)	0.3585 (4)	0.0456 (11)	
O1	0.1425 (4)	0.6937 (4)	0.3365 (3)	0.0488 (10)	
O2	0.2724 (4)	0.7142 (4)	0.2302 (4)	0.0522 (10)	
O3	0.6255 (4)	1.0193 (3)	0.5933 (3)	0.0384 (8)	
O4	0.5990 (4)	0.8317 (3)	0.5899 (4)	0.0526 (11)	
O5	0.5617 (4)	0.8922 (3)	0.3554 (3)	0.0421 (8)	
O6	0.3488 (4)	0.8965 (3)	0.6021 (4)	0.0478 (9)	

### Atomic displacement parameters (Å^2^)

**Table:**

	*U*^11^	*U*^22^	*U*^33^	*U*^12^	*U*^13^	*U*^23^
Gd1	0.03152 (16)	0.02485 (15)	0.04068 (18)	0.01156 (11)	0.00743 (11)	0.01632 (11)
C1	0.053 (4)	0.044 (3)	0.067 (4)	0.025 (3)	0.016 (3)	0.014 (3)
C2	0.080 (5)	0.068 (5)	0.063 (4)	0.051 (4)	0.012 (4)	0.006 (4)
C3	0.099 (6)	0.047 (4)	0.060 (4)	0.049 (4)	−0.006 (4)	0.000 (3)
C4	0.084 (5)	0.035 (3)	0.056 (4)	0.030 (3)	−0.009 (4)	0.006 (3)
C5	0.054 (3)	0.029 (3)	0.041 (3)	0.020 (2)	−0.010 (3)	0.009 (2)
C6	0.034 (3)	0.034 (3)	0.039 (3)	0.015 (2)	0.005 (2)	0.017 (2)
C7	0.038 (3)	0.036 (3)	0.052 (3)	0.023 (2)	0.007 (2)	0.013 (2)
C8	0.051 (4)	0.059 (4)	0.089 (5)	0.027 (3)	0.026 (4)	0.044 (4)
C9	0.050 (4)	0.068 (5)	0.130 (8)	0.026 (4)	0.037 (5)	0.054 (5)
C10	0.042 (4)	0.079 (5)	0.133 (8)	0.031 (4)	0.009 (5)	0.042 (5)
C11	0.050 (4)	0.103 (6)	0.088 (6)	0.040 (4)	−0.001 (4)	0.038 (5)
C12	0.044 (3)	0.070 (4)	0.049 (3)	0.032 (3)	0.008 (3)	0.024 (3)
C13	0.041 (3)	0.026 (2)	0.043 (3)	0.013 (2)	0.005 (2)	0.011 (2)
C14	0.048 (3)	0.043 (3)	0.037 (3)	0.019 (3)	0.005 (2)	0.017 (2)
C15	0.042 (3)	0.084 (5)	0.042 (3)	0.020 (3)	0.012 (3)	0.026 (3)
C16	0.035 (3)	0.109 (7)	0.066 (5)	0.025 (4)	−0.001 (3)	0.026 (4)
C17	0.064 (5)	0.079 (5)	0.056 (4)	0.030 (4)	−0.017 (4)	0.019 (4)
C18	0.083 (6)	0.080 (5)	0.046 (4)	0.029 (4)	0.011 (4)	0.031 (4)
C19	0.056 (4)	0.058 (4)	0.051 (4)	0.012 (3)	0.015 (3)	0.030 (3)
C20	0.035 (3)	0.035 (3)	0.048 (3)	0.018 (2)	0.017 (2)	0.020 (2)
C21	0.049 (3)	0.046 (3)	0.054 (3)	0.031 (3)	0.025 (3)	0.026 (3)
C22	0.066 (4)	0.045 (3)	0.069 (4)	0.027 (3)	0.040 (3)	0.029 (3)
C23	0.099 (6)	0.073 (5)	0.085 (5)	0.059 (5)	0.066 (5)	0.052 (4)
C24	0.092 (6)	0.079 (5)	0.057 (4)	0.051 (5)	0.038 (4)	0.027 (4)
C25	0.078 (5)	0.065 (4)	0.046 (4)	0.032 (4)	0.023 (3)	0.010 (3)
C26	0.050 (3)	0.056 (4)	0.060 (4)	0.023 (3)	0.031 (3)	0.027 (3)
C27	0.053 (4)	0.061 (4)	0.089 (5)	0.028 (3)	0.030 (4)	0.050 (4)
C28	0.065 (5)	0.075 (5)	0.107 (6)	0.025 (4)	0.032 (4)	0.068 (5)
C29	0.085 (6)	0.058 (5)	0.107 (7)	0.006 (4)	0.019 (5)	0.060 (5)
C30	0.092 (6)	0.037 (4)	0.083 (6)	0.007 (4)	−0.004 (5)	0.033 (4)
C31	0.056 (4)	0.028 (3)	0.052 (3)	0.011 (2)	−0.007 (3)	0.021 (2)
F1	0.078 (3)	0.061 (2)	0.087 (3)	0.004 (2)	0.048 (2)	0.025 (2)
F2	0.111 (4)	0.098 (4)	0.057 (3)	0.024 (3)	0.033 (3)	0.000 (3)
F3	0.070 (3)	0.169 (5)	0.069 (3)	0.055 (3)	0.025 (2)	0.071 (3)
F4	0.072 (3)	0.148 (5)	0.253 (8)	0.052 (3)	0.089 (4)	0.135 (6)
F5	0.092 (5)	0.272 (10)	0.123 (6)	0.029 (5)	0.033 (4)	0.099 (6)
F6	0.151 (7)	0.295 (12)	0.128 (7)	0.030 (7)	0.016 (5)	0.120 (8)
N1	0.038 (3)	0.038 (2)	0.065 (3)	0.013 (2)	0.009 (2)	0.031 (2)
N2	0.043 (3)	0.033 (2)	0.055 (3)	0.018 (2)	0.005 (2)	0.018 (2)
O1	0.042 (2)	0.055 (2)	0.044 (2)	0.0152 (18)	0.0094 (17)	0.0274 (19)
O2	0.040 (2)	0.058 (3)	0.047 (2)	0.0221 (19)	0.0079 (18)	0.013 (2)
O3	0.0357 (18)	0.0307 (17)	0.048 (2)	0.0166 (15)	0.0074 (16)	0.0200 (16)
O4	0.044 (2)	0.0254 (18)	0.068 (3)	0.0106 (16)	−0.0058 (19)	0.0200 (18)
O5	0.041 (2)	0.0355 (19)	0.053 (2)	0.0166 (16)	0.0211 (17)	0.0215 (17)
O6	0.057 (2)	0.034 (2)	0.052 (2)	0.0167 (18)	0.0257 (19)	0.0200 (18)

### Geometric parameters (Å, °)

**Table:**

Gd1—O6	2.364 (4)	C13—C14	1.489 (8)
Gd1—O3^i^	2.378 (3)	C14—C15	1.377 (9)
Gd1—O5	2.380 (4)	C14—C19	1.409 (8)
Gd1—O2	2.419 (4)	C15—F5	1.279 (9)
Gd1—O4	2.482 (4)	C15—C16	1.357 (9)
Gd1—O1	2.495 (4)	C16—C17	1.347 (12)
Gd1—N1	2.567 (4)	C16—H16	0.9300
Gd1—N2	2.585 (5)	C17—C18	1.375 (12)
Gd1—O3	2.692 (4)	C17—H17	0.9300
Gd1—C13	2.806 (5)	C18—C19	1.345 (10)
Gd1—C6	2.942 (5)	C18—F6	1.350 (11)
Gd1—Gd1^i^	4.0615 (12)	C19—H19	0.9300
C1—N2	1.319 (8)	C20—O5	1.239 (6)
C1—C2	1.395 (9)	C20—O6^i^	1.253 (6)
C1—H1	0.9300	C20—C21	1.511 (8)
C2—C3	1.322 (12)	C21—C22	1.369 (8)
C2—H2	0.9300	C21—C26	1.397 (9)
C3—C4	1.363 (12)	C22—F1	1.335 (8)
C3—H3	0.9300	C22—C23	1.386 (10)
C4—C5	1.382 (9)	C23—C24	1.380 (11)
C4—H4	0.9300	C23—H23	0.9300
C5—N2	1.342 (7)	C24—C25	1.339 (10)
C5—C31	1.467 (10)	C24—H24	0.9300
C6—O4	1.237 (6)	C25—F2	1.352 (8)
C6—O3	1.261 (6)	C25—C26	1.399 (9)
C6—C7	1.505 (7)	C26—H26	0.9300
C7—C8	1.371 (9)	C27—N1	1.330 (9)
C7—C12	1.383 (9)	C27—C28	1.352 (9)
C8—C9	1.389 (10)	C27—H27	0.9300
C8—H8	0.9300	C28—C29	1.324 (13)
C9—C10	1.309 (13)	C28—H28	0.9300
C9—F4	1.335 (9)	C29—C30	1.384 (14)
C10—C11	1.409 (13)	C29—H29	0.9300
C10—H10	0.9300	C30—C31	1.389 (9)
C11—C12	1.380 (9)	C30—H30	0.9300
C11—H11	0.9300	C31—N1	1.352 (8)
C12—F3	1.325 (8)	O3—Gd1^i^	2.378 (3)
C13—O1	1.258 (7)	O6—C20^i^	1.253 (6)
C13—O2	1.254 (7)		
			
O6—Gd1—O3^i^	75.83 (13)	C9—C8—C7	118.9 (7)
O6—Gd1—O5	132.95 (13)	C9—C8—H8	120.5
O3^i^—Gd1—O5	74.27 (13)	C7—C8—H8	120.5
O6—Gd1—O2	132.75 (15)	C10—C9—F4	118.7 (8)
O3^i^—Gd1—O2	78.28 (14)	C10—C9—C8	122.7 (8)
O5—Gd1—O2	74.17 (14)	F4—C9—C8	118.6 (8)
O6—Gd1—O4	84.95 (15)	C9—C10—C11	120.5 (7)
O3^i^—Gd1—O4	123.14 (12)	C9—C10—H10	119.8
O5—Gd1—O4	81.99 (14)	C11—C10—H10	119.8
O2—Gd1—O4	142.06 (15)	C12—C11—C10	117.1 (8)
O6—Gd1—O1	84.39 (15)	C12—C11—H11	121.4
O3^i^—Gd1—O1	81.23 (13)	C10—C11—H11	121.4
O5—Gd1—O1	125.10 (13)	F3—C12—C7	119.0 (5)
O2—Gd1—O1	52.89 (14)	F3—C12—C11	118.8 (6)
O4—Gd1—O1	149.72 (13)	C7—C12—C11	122.2 (7)
O6—Gd1—N1	79.37 (15)	O1—C13—O2	121.3 (5)
O3^i^—Gd1—N1	144.99 (15)	O1—C13—C14	119.4 (5)
O5—Gd1—N1	140.06 (15)	O2—C13—C14	119.2 (5)
O2—Gd1—N1	101.82 (16)	O1—C13—Gd1	62.8 (3)
O4—Gd1—N1	78.17 (14)	O2—C13—Gd1	59.3 (3)
O1—Gd1—N1	72.04 (14)	C14—C13—Gd1	168.3 (4)
O6—Gd1—N2	138.74 (15)	C15—C14—C19	114.5 (6)
O3^i^—Gd1—N2	145.41 (15)	C15—C14—C13	125.5 (6)
O5—Gd1—N2	78.19 (14)	C19—C14—C13	120.0 (6)
O2—Gd1—N2	74.34 (15)	F5—C15—C16	114.6 (7)
O4—Gd1—N2	72.15 (14)	F5—C15—C14	121.2 (6)
O1—Gd1—N2	98.28 (15)	C16—C15—C14	124.2 (7)
N1—Gd1—N2	62.87 (17)	C17—C16—C15	120.1 (7)
O6—Gd1—O3	70.83 (13)	C17—C16—H16	119.9
O3^i^—Gd1—O3	73.72 (12)	C15—C16—H16	119.9
O5—Gd1—O3	66.40 (12)	C16—C17—C18	117.8 (6)
O2—Gd1—O3	136.31 (13)	C16—C17—H17	121.1
O4—Gd1—O3	49.42 (11)	C18—C17—H17	121.1
O1—Gd1—O3	148.18 (13)	C19—C18—F6	115.1 (8)
N1—Gd1—O3	120.33 (13)	C19—C18—C17	122.5 (7)
N2—Gd1—O3	113.49 (13)	F6—C18—C17	122.4 (8)
O6—Gd1—C13	108.05 (16)	C18—C19—C14	120.8 (7)
O3^i^—Gd1—C13	76.10 (14)	C18—C19—H19	119.6
O5—Gd1—C13	98.99 (15)	C14—C19—H19	119.6
O2—Gd1—C13	26.47 (16)	O5—C20—O6^i^	126.5 (5)
O4—Gd1—C13	159.67 (14)	O5—C20—C21	115.8 (5)
O1—Gd1—C13	26.63 (15)	O6^i^—C20—C21	117.8 (5)
N1—Gd1—C13	88.73 (16)	C22—C21—C26	119.4 (6)
N2—Gd1—C13	88.09 (15)	C22—C21—C20	124.0 (5)
O3—Gd1—C13	149.07 (13)	C26—C21—C20	116.6 (5)
O6—Gd1—C6	80.23 (15)	F1—C22—C23	118.8 (6)
O3^i^—Gd1—C6	98.81 (13)	F1—C22—C21	120.7 (6)
O5—Gd1—C6	69.55 (14)	C23—C22—C21	120.4 (7)
O2—Gd1—C6	142.89 (15)	C24—C23—C22	120.9 (7)
O4—Gd1—C6	24.53 (12)	C24—C23—H23	119.6
O1—Gd1—C6	164.08 (15)	C22—C23—H23	119.6
N1—Gd1—C6	100.90 (14)	C25—C24—C23	118.1 (7)
N2—Gd1—C6	90.66 (15)	C25—C24—H24	120.9
O3—Gd1—C6	25.36 (12)	C23—C24—H24	120.9
C13—Gd1—C6	168.47 (16)	F2—C25—C24	119.3 (6)
O6—Gd1—Gd1^i^	68.84 (9)	F2—C25—C26	117.5 (7)
O3^i^—Gd1—Gd1^i^	39.52 (8)	C24—C25—C26	123.2 (7)
O5—Gd1—Gd1^i^	64.90 (9)	C25—C26—C21	117.9 (6)
O2—Gd1—Gd1^i^	111.12 (11)	C25—C26—H26	121.0
O4—Gd1—Gd1^i^	83.62 (8)	C21—C26—H26	121.0
O1—Gd1—Gd1^i^	118.30 (10)	N1—C27—C28	123.7 (8)
N1—Gd1—Gd1^i^	144.52 (12)	N1—C27—H27	118.1
N2—Gd1—Gd1^i^	138.26 (11)	C28—C27—H27	118.1
O3—Gd1—Gd1^i^	34.20 (7)	C29—C28—C27	119.4 (9)
C13—Gd1—Gd1^i^	115.34 (11)	C29—C28—H28	120.3
C6—Gd1—Gd1^i^	59.38 (10)	C27—C28—H28	120.3
N2—C1—C2	123.4 (7)	C28—C29—C30	119.6 (7)
N2—C1—H1	118.3	C28—C29—H29	120.2
C2—C1—H1	118.3	C30—C29—H29	120.2
C3—C2—C1	118.2 (8)	C29—C30—C31	119.2 (8)
C3—C2—H2	120.9	C29—C30—H30	120.4
C1—C2—H2	120.9	C31—C30—H30	120.4
C2—C3—C4	120.1 (7)	N1—C31—C30	120.0 (8)
C2—C3—H3	119.9	N1—C31—C5	116.6 (5)
C4—C3—H3	119.9	C30—C31—C5	123.4 (7)
C3—C4—C5	119.6 (7)	C27—N1—C31	118.1 (5)
C3—C4—H4	120.2	C27—N1—Gd1	120.0 (4)
C5—C4—H4	120.2	C31—N1—Gd1	120.8 (4)
N2—C5—C4	121.1 (7)	C1—N2—C5	117.6 (5)
N2—C5—C31	116.7 (5)	C1—N2—Gd1	121.2 (4)
C4—C5—C31	122.2 (6)	C5—N2—Gd1	121.2 (4)
O4—C6—O3	120.8 (5)	C13—O1—Gd1	90.6 (3)
O4—C6—C7	119.9 (4)	C13—O2—Gd1	94.2 (3)
O3—C6—C7	119.2 (4)	C6—O3—Gd1^i^	163.0 (3)
O4—C6—Gd1	56.4 (3)	C6—O3—Gd1	88.5 (3)
O3—C6—Gd1	66.2 (3)	Gd1^i^—O3—Gd1	106.28 (12)
C7—C6—Gd1	162.8 (4)	C6—O4—Gd1	99.0 (3)
C8—C7—C12	118.6 (6)	C20—O5—Gd1	135.6 (3)
C8—C7—C6	119.9 (5)	C20^i^—O6—Gd1	133.6 (3)
C12—C7—C6	121.4 (5)		
			
O6—Gd1—O1—C13	153.0 (3)	O5—Gd1—C6—O4	−117.5 (4)
O3^i^—Gd1—O1—C13	76.5 (3)	O2—Gd1—C6—O4	−104.8 (4)
O5—Gd1—O1—C13	12.9 (4)	O1—Gd1—C6—O4	84.1 (6)
O2—Gd1—O1—C13	−5.4 (3)	N1—Gd1—C6—O4	22.1 (4)
O4—Gd1—O1—C13	−137.2 (4)	N2—Gd1—C6—O4	−40.3 (4)
N1—Gd1—O1—C13	−126.4 (4)	O3—Gd1—C6—O4	164.6 (6)
N2—Gd1—O1—C13	−68.5 (3)	C13—Gd1—C6—O4	−123.9 (7)
O3—Gd1—O1—C13	114.6 (3)	Gd1^i^—Gd1—C6—O4	170.3 (4)
C6—Gd1—O1—C13	167.9 (4)	O6—Gd1—C6—O3	−65.4 (3)
Gd1^i^—Gd1—O1—C13	90.7 (3)	O3^i^—Gd1—C6—O3	8.5 (4)
O6—Gd1—O2—C13	−24.6 (4)	O5—Gd1—C6—O3	77.9 (3)
O3^i^—Gd1—O2—C13	−82.4 (3)	O2—Gd1—C6—O3	90.6 (4)
O5—Gd1—O2—C13	−159.2 (4)	O4—Gd1—C6—O3	−164.6 (6)
O4—Gd1—O2—C13	147.7 (3)	O1—Gd1—C6—O3	−80.5 (6)
O1—Gd1—O2—C13	5.4 (3)	N1—Gd1—C6—O3	−142.5 (3)
N1—Gd1—O2—C13	61.8 (4)	N2—Gd1—C6—O3	155.1 (3)
N2—Gd1—O2—C13	118.9 (4)	C13—Gd1—C6—O3	71.5 (8)
O3—Gd1—O2—C13	−133.2 (3)	Gd1^i^—Gd1—C6—O3	5.7 (3)
C6—Gd1—O2—C13	−171.5 (3)	O6—Gd1—C6—C7	−177.5 (12)
Gd1^i^—Gd1—O2—C13	−104.8 (3)	O3^i^—Gd1—C6—C7	−103.6 (12)
O6—Gd1—O3—C6	108.4 (3)	O5—Gd1—C6—C7	−34.2 (12)
O3^i^—Gd1—O3—C6	−171.3 (4)	O2—Gd1—C6—C7	−21.5 (13)
O5—Gd1—O3—C6	−91.7 (3)	O4—Gd1—C6—C7	83.3 (12)
O2—Gd1—O3—C6	−119.1 (3)	O1—Gd1—C6—C7	167.4 (10)
O4—Gd1—O3—C6	8.3 (3)	N1—Gd1—C6—C7	105.4 (12)
O1—Gd1—O3—C6	149.2 (3)	N2—Gd1—C6—C7	43.0 (12)
N1—Gd1—O3—C6	43.8 (4)	O3—Gd1—C6—C7	−112.1 (13)
N2—Gd1—O3—C6	−27.4 (3)	C13—Gd1—C6—C7	−40.6 (16)
C13—Gd1—O3—C6	−158.3 (4)	Gd1^i^—Gd1—C6—C7	−106.4 (12)
Gd1^i^—Gd1—O3—C6	−171.3 (4)	O4—C6—C7—C8	120.0 (7)
O6—Gd1—O3—Gd1^i^	−80.30 (16)	O3—C6—C7—C8	−56.7 (8)
O3^i^—Gd1—O3—Gd1^i^	0.0	Gd1—C6—C7—C8	47.2 (14)
O5—Gd1—O3—Gd1^i^	79.60 (15)	O4—C6—C7—C12	−57.5 (8)
O2—Gd1—O3—Gd1^i^	52.2 (2)	O3—C6—C7—C12	125.8 (6)
O4—Gd1—O3—Gd1^i^	179.6 (2)	Gd1—C6—C7—C12	−130.3 (11)
O1—Gd1—O3—Gd1^i^	−39.5 (3)	C12—C7—C8—C9	0.6 (10)
N1—Gd1—O3—Gd1^i^	−144.87 (17)	C6—C7—C8—C9	−177.0 (6)
N2—Gd1—O3—Gd1^i^	143.94 (16)	C7—C8—C9—C10	−2.1 (13)
C13—Gd1—O3—Gd1^i^	13.0 (4)	C7—C8—C9—F4	178.9 (7)
C6—Gd1—O3—Gd1^i^	171.3 (4)	F4—C9—C10—C11	−179.4 (8)
O6—Gd1—O4—C6	−77.6 (4)	C8—C9—C10—C11	1.6 (15)
O3^i^—Gd1—O4—C6	−8.2 (4)	C9—C10—C11—C12	0.3 (14)
O5—Gd1—O4—C6	57.1 (4)	C10—C11—C12—F3	178.5 (8)
O2—Gd1—O4—C6	108.1 (4)	C10—C11—C12—C7	−1.8 (13)
O1—Gd1—O4—C6	−147.3 (4)	C8—C7—C12—F3	−178.9 (6)
N1—Gd1—O4—C6	−157.8 (4)	C6—C7—C12—F3	−1.4 (10)
N2—Gd1—O4—C6	137.2 (4)	C8—C7—C12—C11	1.4 (11)
O3—Gd1—O4—C6	−8.6 (3)	C6—C7—C12—C11	178.9 (7)
C13—Gd1—O4—C6	151.4 (5)	Gd1—O2—C13—O1	−10.1 (6)
Gd1^i^—Gd1—O4—C6	−8.4 (4)	Gd1—O2—C13—C14	166.6 (4)
O6—Gd1—O5—C20	−43.1 (6)	Gd1—O1—C13—O2	9.7 (5)
O3^i^—Gd1—O5—C20	9.3 (5)	Gd1—O1—C13—C14	−166.9 (4)
O2—Gd1—O5—C20	91.3 (5)	O6—Gd1—C13—O2	161.3 (3)
O4—Gd1—O5—C20	−118.5 (5)	O3^i^—Gd1—C13—O2	91.5 (3)
O1—Gd1—O5—C20	76.2 (5)	O5—Gd1—C13—O2	20.3 (3)
N1—Gd1—O5—C20	−179.1 (5)	O4—Gd1—C13—O2	−71.0 (6)
N2—Gd1—O5—C20	168.1 (5)	O1—Gd1—C13—O2	−170.3 (5)
O3—Gd1—O5—C20	−69.5 (5)	N1—Gd1—C13—O2	−120.3 (3)
C13—Gd1—O5—C20	82.0 (5)	N2—Gd1—C13—O2	−57.5 (3)
C6—Gd1—O5—C20	−96.7 (5)	O3—Gd1—C13—O2	78.6 (4)
Gd1^i^—Gd1—O5—C20	−31.8 (5)	C6—Gd1—C13—O2	26.3 (9)
O3^i^—Gd1—O6—C20^i^	−43.7 (5)	Gd1^i^—Gd1—C13—O2	86.7 (3)
O5—Gd1—O6—C20^i^	8.2 (6)	O6—Gd1—C13—O1	−28.4 (3)
O2—Gd1—O6—C20^i^	−102.4 (5)	O3^i^—Gd1—C13—O1	−98.2 (3)
O4—Gd1—O6—C20^i^	82.3 (5)	O5—Gd1—C13—O1	−169.4 (3)
O1—Gd1—O6—C20^i^	−126.0 (5)	O2—Gd1—C13—O1	170.3 (5)
N1—Gd1—O6—C20^i^	161.2 (5)	O4—Gd1—C13—O1	99.4 (6)
N2—Gd1—O6—C20^i^	137.8 (5)	N1—Gd1—C13—O1	50.0 (3)
O3—Gd1—O6—C20^i^	33.7 (5)	N2—Gd1—C13—O1	112.8 (3)
C13—Gd1—O6—C20^i^	−113.7 (5)	O3—Gd1—C13—O1	−111.0 (4)
C6—Gd1—O6—C20^i^	58.1 (5)	C6—Gd1—C13—O1	−163.3 (6)
Gd1^i^—Gd1—O6—C20^i^	−2.8 (5)	Gd1^i^—Gd1—C13—O1	−103.0 (3)
O6—Gd1—N1—C27	18.7 (5)	O6—Gd1—C13—C14	75 (2)
O3^i^—Gd1—N1—C27	−26.7 (6)	O3^i^—Gd1—C13—C14	6(2)
O5—Gd1—N1—C27	167.5 (5)	O5—Gd1—C13—C14	−66 (2)
O2—Gd1—N1—C27	−113.1 (5)	O2—Gd1—C13—C14	−86 (2)
O4—Gd1—N1—C27	105.7 (5)	O4—Gd1—C13—C14	−157 (2)
O1—Gd1—N1—C27	−68.8 (5)	O1—Gd1—C13—C14	104 (2)
N2—Gd1—N1—C27	−178.5 (5)	N1—Gd1—C13—C14	154 (2)
O3—Gd1—N1—C27	78.9 (5)	N2—Gd1—C13—C14	−143 (2)
C13—Gd1—N1—C27	−90.0 (5)	O3—Gd1—C13—C14	−7(2)
C6—Gd1—N1—C27	96.5 (5)	C6—Gd1—C13—C14	−60 (3)
Gd1^i^—Gd1—N1—C27	45.0 (6)	Gd1^i^—Gd1—C13—C14	1(2)
O6—Gd1—N1—C31	−174.0 (4)	O2—C13—C14—C15	166.7 (7)
O3^i^—Gd1—N1—C31	140.6 (4)	O1—C13—C14—C15	−16.6 (9)
O5—Gd1—N1—C31	−25.2 (5)	Gd1—C13—C14—C15	−114 (2)
O2—Gd1—N1—C31	54.2 (4)	O2—C13—C14—C19	−15.2 (8)
O4—Gd1—N1—C31	−87.0 (4)	O1—C13—C14—C19	161.6 (6)
O1—Gd1—N1—C31	98.5 (4)	Gd1—C13—C14—C19	64 (2)
N2—Gd1—N1—C31	−11.1 (4)	C19—C14—C15—F5	−178.7 (9)
O3—Gd1—N1—C31	−113.8 (4)	C13—C14—C15—F5	−0.4 (13)
C13—Gd1—N1—C31	77.4 (4)	C19—C14—C15—C16	0.9 (12)
C6—Gd1—N1—C31	−96.2 (4)	C13—C14—C15—C16	179.1 (8)
Gd1^i^—Gd1—N1—C31	−147.7 (3)	F5—C15—C16—C17	178.4 (10)
O6—Gd1—N2—C1	−148.1 (4)	C14—C15—C16—C17	−1.2 (15)
O3^i^—Gd1—N2—C1	34.4 (6)	C15—C16—C17—C18	0.8 (14)
O5—Gd1—N2—C1	−3.3 (4)	C16—C17—C18—C19	−0.3 (14)
O2—Gd1—N2—C1	73.4 (5)	C16—C17—C18—F6	178.4 (10)
O4—Gd1—N2—C1	−88.6 (5)	F6—C18—C19—C14	−178.7 (9)
O1—Gd1—N2—C1	121.0 (5)	C17—C18—C19—C14	0.1 (13)
N1—Gd1—N2—C1	−174.1 (5)	C15—C14—C19—C18	−0.3 (11)
O3—Gd1—N2—C1	−60.8 (5)	C13—C14—C19—C18	−178.7 (7)
C13—Gd1—N2—C1	96.3 (5)	Gd1—O5—C20—O6^i^	48.8 (8)
C6—Gd1—N2—C1	−72.2 (5)	Gd1—O5—C20—C21	−130.3 (5)
Gd1^i^—Gd1—N2—C1	−31.0 (5)	O5—C20—C21—C22	−147.5 (6)
O6—Gd1—N2—C5	30.7 (5)	O6^i^—C20—C21—C22	33.3 (8)
O3^i^—Gd1—N2—C5	−146.7 (4)	O5—C20—C21—C26	34.0 (7)
O5—Gd1—N2—C5	175.5 (4)	O6^i^—C20—C21—C26	−145.3 (5)
O2—Gd1—N2—C5	−107.8 (4)	C26—C21—C22—F1	−177.0 (6)
O4—Gd1—N2—C5	90.3 (4)	C20—C21—C22—F1	4.5 (9)
O1—Gd1—N2—C5	−60.1 (4)	C26—C21—C22—C23	−0.4 (10)
N1—Gd1—N2—C5	4.7 (4)	C20—C21—C22—C23	−178.9 (6)
O3—Gd1—N2—C5	118.0 (4)	F1—C22—C23—C24	179.0 (7)
C13—Gd1—N2—C5	−84.8 (4)	C21—C22—C23—C24	2.3 (11)
C6—Gd1—N2—C5	106.7 (4)	C22—C23—C24—C25	−2.3 (11)
Gd1^i^—Gd1—N2—C5	147.8 (3)	C23—C24—C25—F2	−179.5 (7)
C5—N2—C1—C2	−1.8 (9)	C23—C24—C25—C26	0.3 (12)
Gd1—N2—C1—C2	177.1 (5)	C22—C21—C26—C25	−1.5 (9)
N2—C1—C2—C3	2.5 (11)	C20—C21—C26—C25	177.1 (6)
C1—C2—C3—C4	−2.2 (11)	C24—C25—C26—C21	1.6 (11)
C2—C3—C4—C5	1.4 (11)	F2—C25—C26—C21	−178.6 (6)
C1—N2—C5—C4	0.9 (8)	C31—N1—C27—C28	−0.6 (10)
Gd1—N2—C5—C4	−178.0 (4)	Gd1—N1—C27—C28	167.0 (6)
C1—N2—C5—C31	−179.9 (5)	N1—C27—C28—C29	−1.3 (13)
Gd1—N2—C5—C31	1.2 (6)	C27—C28—C29—C30	2.2 (13)
C3—C4—C5—N2	−0.7 (9)	C28—C29—C30—C31	−1.2 (13)
C3—C4—C5—C31	−179.9 (6)	C27—N1—C31—C30	1.5 (9)
Gd1—O4—C6—O3	16.4 (6)	Gd1—N1—C31—C30	−166.0 (5)
Gd1—O4—C6—C7	−160.3 (5)	C27—N1—C31—C5	−176.1 (6)
Gd1^i^—O3—C6—O4	−165.2 (9)	Gd1—N1—C31—C5	16.4 (6)
Gd1—O3—C6—O4	−14.9 (6)	C29—C30—C31—N1	−0.6 (11)
Gd1^i^—O3—C6—C7	11.4 (16)	C29—C30—C31—C5	176.8 (7)
Gd1—O3—C6—C7	161.8 (5)	N2—C5—C31—N1	−11.4 (7)
Gd1^i^—O3—C6—Gd1	−150.3 (12)	C4—C5—C31—N1	167.8 (5)
O6—Gd1—C6—O4	99.2 (4)	N2—C5—C31—C30	171.1 (6)
O3^i^—Gd1—C6—O4	173.1 (4)	C4—C5—C31—C30	−9.7 (9)

Symmetry codes: (i) −*x*+1, −*y*+2, −*z*+1.
